# A Mixed Methods Investigation of the Prevalence and Influencing Factors of Compassion Fatigue among Midwives in Different Areas of China

This article has been retracted.

**DOI:** 10.1155/2022/1815417

**Published:** 2022-10-12

**Authors:** Xin Liang, Ping Yuan, Xingyan Su, Yuanyuan Xing, Kejiao Qiang, Zumei Gao, Jun Wang

**Affiliations:** ^1^Nanyang The First People's Hospital, Nanyang 473000, China; ^2^The Second Affiliated Hospital of Chongqing Medical University, Chongqing 400010, China; ^3^The Central Hospital Of Enshi Tujia And Miao Autonomous Prefecture, Enshi 445000, China; ^4^The Seventh Affiliated Hospital, Sun Yat-sen University, Shenzhen 518107, China; ^5^The First Affiliated Hospital of Yangtze University, Jingzhou 434020, China; ^6^West China Hospital of Sichuan University, Chengdu 610000, China

## Abstract

**Objective:**

Exploring the influencing factors of compassion fatigue among midwives to prevent compassion fatigue from occurring and improve their mental health.

**Methods:**

A method integrating the quantitative research method and qualitative research method is used. For the quantitative research, a cross-sectional study was carried out. State-run hospitals from three economic areas in China were selected as investigation scope from June 2018 to May 2021. A total of 515 midwives were chosen randomly from three economic areas. SPSS 22.0 was used for data cleaning and statistical description and analysis. The influencing factors of compassion fatigue among midwives were analyzed by fitting these two-level logistic models. For qualitative research, purposive sampling and maximum variation strategy were used to select midwives with mild or above compassion fatigue in the questionnaire survey. Field study and interviews were used to collect data.

**Results:**

The results in the quantitative research showed that 515 valid questionnaires were received with 82.14% of midwives whose compassion fatigue were moderate or above. Multilevel statistical model analysis demonstrated that hospital level, children situation, area, working atmosphere, experiences of traumatic delivery, sleep quality, and social support level had impacts on the degree of midwives' compassion fatigue (*p* < 0.05). The result in the qualitative research showed that 34 midwives were interviewed, and 7 topic ideas were refined.

**Conclusion:**

Overall, the incidence of compassion fatigue among midwives is high. Risk factors influencing the degree of midwives' compassion fatigue include lower social support, disharmonious working atmosphere, toddler situation, huge workload, experiences of traumatic delivery, and poor quality of sleep.

## 1. Introduction

*Medium and long term talent development plan of medicine and health 2011-2020* states that it is indispensable to improve team construction of midwives and create new policy, society, and working and living environment to develop talents [1]. Improve midwives' team construction is beneficial to maternal and fetal health and guarantees the high quality of care [2]. A slice of research [3, 4] has examined that traumatic stress influences mental health of midwives and further affects team construction, wherein the most common traumatic stress is traumatic delivery. 78.7% to 84% of midwives experienced at least one traumatic delivery in their works. Traumatic delivery is defined as a series of events that introduce threatening injury or even the risk of death to fetus and puerpera during labor or after a few hours postpartum, such as stillbirth, shoulder dystocia, three-degree perineal laceration, and postpartum hemorrhage. Furthermore, traumatic delivery brings psychological trauma to puerpera and their families and causes traumatic stress reactions among midwives [5–8]. With the opening of two-child policy and the development of birth attendance in China, people put forward more and more demands with the ability of midwives, meanwhile, the workload and work strength of midwives are soaring. Midwives should not only be professional but also take responsibility for caring mental health of puerperae. Due to high risks and heavy workloads, midwives always encounter situations full of stressors during clinical works, which increases the incidence of compassion fatigue [9]. It not only affects the physical and mental health of midwives but also affects the quality of midwifery technology and team building. Their working status, mood, and attitude will also directly affect the physical and mental health and safety of pregnant women. At present, the research on compassion fatigue of midwives abroad is relatively mature, and it has gradually expanded to the study of the connotation and influencing factors of compassion fatigue, intervention implementation, and effect evaluation. In China, only cross-sectional research on midwives' job burnout is conducted, while job burnout is one of the three factors of compassion fatigue. At the same time, due to cultural differences in China and abroad and different hospital management policies in my country, such as different employment forms, leadership styles, and hospital levels, it may be a risk factor for midwives to reduce compassion fatigue. Therefore, it is necessary to analyze the status quo of compassion fatigue of midwives in our country and its influencing factors.

Adams et al.' research [10] states that low social support can worse compassion fatigue among midwives, accordingly, deeply understanding the influencing factors of social support can provide a basis for increase the level of social support. Meanwhile, because of a vast territory and unequal distribution of medical resources in China, influences of regional disparities on midwives' compassion fatigue are worthy of study. In addition, the assessment of physical and mental health of midwives should not only focus on their status but also pour attention into their experiences, where in the diversity of experiences is mostly mutual communication based. Thus, explanatory sequential mixed methods design was used to research midwives from different hospitals in different provinces. Multilevel samples were representative, which can verify and supplement quantitative research and improve excessive dependence on qualities of researchers in qualitative research, in order to make up for the lack of in-depth and dynamic emotional research on the research objects, the current research mostly uses quantitative research.

## 2. Methods

### 2.1. Research Questions

Four specific research questions were asked: (1) are there any differences among midwives from different hospitals in different areas in terms of the degree of compassion fatigue? (2) What are influencing factors of compassion fatigue among midwives? (3) Are midwives more serious than nurses from other departments in terms of the degree of compassion fatigue? (4) How to integrate quantitative research with qualitative research effectively to make a clear and accurate analysis of influencing factors of compassion fatigue among midwives?

### 2.2. Design

This study used explanatory sequential mixed methods design, including two stages. The first stage was collecting quantitative data and then making analysis. Qualitative research [11] was conducted by using the results obtained from the first stage, followed by explaining research results. Cross-sectional study was used in quantitative research. Qualitative research used field study to collect data, including field observation, fieldwork notes, and semistructured and in-depth interviews.

### 2.3. Participants and procedure

Convenient sampling was used to select public hospitals from three economic areas in eastern, central, and western China from June 2018 to May 2021, followed by randomly choosing four provinces from eastern, central, and western China, respectively, in the range of 35 provinces and municipalities in these three economic areas. Once 12 provinces are obtained, 57 hospitals were chosen from secondary, tertiary, and specialized hospitals in selected provinces by using convenient sampling. Then, based on inclusion and exclusion criteria, purposive sampling was used to choose participants (*n* = 515). The inclusion criteria are (1) obtained a Practicing Nurse Certificate and certificate of maternal and infant health care from China, (2) currently works in midwifery, and (3) the working experience is more than 1 year. The exclusion criteria are off-duty midwives because of studying abroad, sick and maternity leave, etc.

Qualitative research used purposive sampling to choose midwives with mild or above compassion fatigue in the questionnaire survey from secondary, tertiary, and specialized hospitals in 6 provinces in quantitative research. To make samples more representative, principle of maximum differentiation was used, to the greatest extent, to select midwives of different ages, titles, hospital levels, areas, and compassion fatigue degree (*n* = 34).

### 2.4. Research tools

1. *General Information Questionnaire*. Questionnaires were self-designed, followed by revising the contents by a panel of experts comprised of 5 associate high or above obstetrics nursing management experts. This questionnaire comprised fundamental information and working environment, the content validity of this questionnaire is 0.92 and Cronbach's *α* is 0.79
2. *Compassion Fatigue Scale*. This scale was developed by Figley and Stamm [12, 13] in 1980s and was used to quantitatively measure compassion fatigue. Each dimension includes 10 items and 30 items in total. Likert 5-class scoring method is used, where 0 indicated strongly unmatched, and 5 indicated strongly matched. The critical values of three dimensions are <37, >27, and >17, respectively. Cronbach's *α* of three dimensions are 0.88, 0.75, and 0.81 separately
3. *Social Support Scale*. This scale was used to measure the degree of social support that an individual receives [13]. This scale includes three dimensions, objective support (three items), subjective support (four items), and support availability (three items). In this scale, low, medium, and high social support are defined as less than score 33, between score 33 and 45, more than score 45, respectively. The test-retest reliability of this scale is 0.92, and the Cronbach's *α* of three dimensions are between 0.89 and 0.94
4. *Interview Outlines*. The questions asked are the following: (1) are there any negative emotions in your work? What are the causes? (2) Does working environment or the style of leader affect your working status? (3) Are there some occasions when the womb is in a crisis caused by adverse events in your work? (4) What are your feelings when faced with pains of puerperae or other appeals in your work? (5) As a midwife, what are your opinions on the supports from family, work, and society? To what extent of these supports? (6) How do you deal with the relationship between family and work? (7) Do you ever desire to quit your job or transfer to other departments during working? (If so, would you mind telling the reasons?)

### 2.5. Data collection methods

Data collection methods in this study included field questionnaire survey and online questionnaire survey.

[1] *Field questionnaire survey*. Field questionnaire survey was in the charge of a researcher who carried out field investigations to surrounding provinces and cities (Hubei, Henan, and Anhui province) of the researcher's area. By the statistics, there were 146 questionnaires issued and 144 were effectively received with effective recovery of 98.63%.

[2] *Online questionnaire survey*. Online questionnaire investigation was made in other provinces and municipalities, and it is indispensable to recruit liaisons from local hospitals. Liaisons should be medical workers and were required to have research basis and obtain at least bachelor's degree. In addition, video training, which should identify the purposes and significance of this research and filling details of scales, was provided for liaisons. Every liaison built a WeChat questionnaire group for their own hospital, and the group administrators would include the researcher, liaison, and people in charge of departments, and group members were research objects. Department heads took responsibility to arrange filling time and supervise the whole process. Liaisons were in charge of distributing the QR code of questionnaire and explaining the investigation purposes, contents, and notice. There were 376 questionnaires issued and 371 were effectively received with effective recovery of 98.67%.

Qualitative researches included in this study are field study and interviews.

[1] *Field Study*. Since field study for in-depth research were feasible in hospitals of Henan, Hubei, and Chongqing provinces, typical and representative objects were selected to conduct on-site and in-depth interviews.

[2] *Interviews*. As for midwives of other provinces, due to the infeasibility of field work, research objects would be chosen according to maximum differences and representativeness to conduct visual interviews, which offset the small sample size and limited representativeness of field study and avoid subjective bias. Under the nursing department's leadership or recommendation, researcher, as a trainee of midwife, participated in the field observation training and studied delivery rooms' working procedures, techniques and regulations systematically. From June 5, 2017 to January 10, 2020, researcher observes the working status of the midwives, and then built trust relationships with them, followed by full participation observation. Besides collecting data by observing and listening, researcher should also record and edit all data observed and then transcribe these data within 24 hours. Appointments with participants who accord with inclusion criteria should be made in advance. Based on the will of the researcher, interview spots could be private, quiet, and comfortable. Every interview would last 30 to 60 minutes. When face-to-face communications were impossible, WeChat video interviews were used. Before the WeChat video interview, the researcher could gain the trust of participants by chatting on WeChat for 10 to 20 days and understand their working and living status in the following 2 to 4 months. The researcher uses WeChat Video to build a face-to-face communication if the interviewees approve. To keep the internet connection available and high video quality, both interviewees and researcher were suggested to choose private and peaceful spots with excellent internet connection.

### 2.6. Data Analysis

EpiData 3.1 was used to build database, and the data were parallel inputted by two individuals, followed by consistency checks. In the data processing and statistical analysis using SPSS 22.0, the measurement data used mean and standard deviation and the count data used frequency and percentage. In terms of single factor analysis, the categorical data used chi-square test and the ranked data used nonparameter Kruskal–Wallis test. Considering that data had a hierarchical structure of hospital and individual, MLwiN 2.30 package was used to analyze the influencing factors of midwives' compassion fatigue by multilevel statistical models. Individuals and hospitals were defined as level 1 and level 2, respectively, followed by fitting two-level logistic models.

Recording and notes need be transcribed within 24 hours after interviews. Then, the transcribed contents should be checked to ensure that all information was true and correct. Content analysis method was adopted in descriptive qualitative research [14], when the subjects were fully determined, interviewer and interviewees should work together to carry on checking process to guarantee the validity of interpretation and data saturation.

## 3. Results

### 3.1. General information comparison

In this study, 515 midwives from 57 hospitals are all females, whose ages are between 23 and 43 (29.84 ± 4.92). Among these midwives, 225 (43.8%) have 1-5 years of working experience, 159 (30.8%) have 6-10 years of working experience, 78 (15.1%) have 11-15 years of working experience, and 53 (10.3%) have more than 15-year experience; 5 midwives (0.9%) only have technical secondary school qualifications, 136 (26.6%) only have college degrees, 370 (71.7%) have bachelor's degrees, and 4 (0.8%) have master's degrees. The sampling situation of investigated hospitals is shown in Table 1.

### 3.2. Single Factor Analysis Results of Midwives' Compassion Fatigue

Single factor analysis results (Table 2) demonstrate that age, marriage situation, hospital level, children situation, numbers of experiences of traumatic delivery, area, working conditions, workload, working environment, level of social support all impact the degree of midwives' compassion fatigue (*P* < 0.05).

### 3.3. Multilevel Statistical Models Analysis of Midwives' Compassion Fatigue

Individuals and hospitals were defined as level 1 and level 2, respectively, followed by fitting two-level logistic models. Results manifest that the variance of level 2 is 0.926 (*P* < 0.05), which means clustering of hospital level exists and the hierarchical structure is not neglected, so multilevel statistical models analysis should be adopted, as is shown in Table 3. Furthermore, some meaningful impact factors from single factor analysis had been introduced into two-level logistic regression models, and analysis had been made for existed models, where unordered categorical variables (hospital, marriage situation, and area) were introduced as dummy variables, and ordered categorical variables were introduced as grouping linear variables and dummy variables, respectively, followed by fitting model 1 and model 2. Ultimately, all ordered categorical variables were introduced as dummy variables by judging whether these two models had statistical significance and linear trend. Assignment method of independent variables is shown in Table 4. Results demonstrate that the level of hospital, area, sleep quality, numbers of experiences of traumatic delivery, children situation, working environment, and the level of social support are all the impact factors of midwives' compassion fatigue (*P* < 0.05), as is shown in Table 5.

### 3.4. Qualitative research

In this study, 34 female midwives, whose mean age was 32.32 ± 4.57, more details are shown in Table 6, were interviewed. The degree of compassion fatigue of them were all mild or above. This research conducted 34 semistructured interviews and transcribed 210,000 words, and then analyzed these transcribed data and field notes to refine themes,, a total of 7 themes, and 24 subthemes. In the date analysis results, field notes were in italics.

#### 3.4.1. Theme 1: Excessive Workloads Lead to Negative Emotions

*Painful*: “The working hours are too long for both day shifts and night shifts and there is no break when working. The whole process is miserable so that I am in no mood to relax myself.” (eyes moist) (ID 2).

*Exhausted*: *Staying up all night with midwife teacher is extremely common. Keeping a good state at every moment is crucial, because there are many deliveries in the night shifts and puerperae are easily to become exhausted on the night.*

*Nervous*: “As a new midwife, I feel nervous with increasing deliveries in recent two years. I have ever thought about quitting because I am worried about making mistakes under large workloads. I am extremely anxious and desire to cry sometimes” (choked up) (M 4).

#### 3.4.2. Theme 2: Incomplete Social Support System

*Misunderstandings Exist*: “What disappoints us is families of puerperae buy gifts to thank for doctors and neglect our efforts after delivery. We do not care about gifts and what we need is recognition (eyes moist).” (ID 29).

*Insufficient Material Needs Support*: “I am working as a midwife for 30 years. I bring in 3000 CNY a month, which is not enough to support my family. We take more risks but obtain less. It would be great if basic hospitals could raise salaries.” (ID 12).

*Desire to Receive Attention: Some midwives were delighted to discuss how to prepare for Nurses Day (May 12^th^). However, after a while, they were told that there was no need for midwives to prepare programs but nurses from obstetrics department can. On hearing this news, all people felt upset without saying a single word.*

*Imbalanced Social Support*: “Workers in western hospitals lack systematic study of midwifery for many years. Though I am assiduous and work for many years, I still see the large gap between us and provincial or municipal hospitals when I take part in provincial or municipal trainings. Many colleagues of mine have never ever left home.” (ID 30).

#### 3.4.3. Theme 3: High Level of Psychological Flexibility

*Head nurse praised a midwife in one regular meeting, who gets divorced but always keeps positive. She needs to send her school-age kid to school by herself regardless of the weather. Instead of complaining the unfair life, she always helps others and participates in charity activities. Meanwhile, when she was praised, she also appreciated the understanding of other colleagues.*

*Positive*: “Perhaps due to young age, I am positive to everything. Each time when I see the newborn in delivery rooms, I feel delighted and confident.” (ID 7).

*Mental Self-Adjustment*: “The ability to self-adjustment is crucial in working. Some negative emotions and things will fade with time, so I do not think too much about that and feel satisfied.” (ID 17).

*Positive Mental Feedback*: “I am working for long and have delivered many newborns. Sometimes when I am shopping or at supermarket, some individuals recognize me and say, ‘it is you who delivered our children', from which I can feel their gratitude. Though it is just a sentence, I still feel delighted and will more assiduous in work.” (ID 5).

#### 3.4.4. Theme 4: Experiences of Traumatic Delivery

*Numbers of Traumatic Delivery*: “I experienced many traumatic deliveries in my 15-year career, which leaves me scarred. Sometimes I feel extremely worried and desire to go to other departments.” (ID 8).

*Severity of Traumatic Delivery*: “Once, there was a puerpera with amniotic fluid embolism (AFE) and we tried our best but failed. I witnessed the death of the woman, which made me extremely painful and struggling for a long time. Even now I still scarcely dare think of that matter.” (ID 27).

*Inappropriate Handling of Superior*: “Once we failed in rescuing a premature baby, the families were very angry and wanted answers. A leader, who did not understand midwifery, rebuked us and tried to find who to blame, which left us with large psychological scars.” (ID 15).

*Negative Handling of Superior: When families make troubles, the head nurse directly hides away. Some midwives are scolded by the families with tears and they do not know how to do but only apologies, which makes worse. They hope that the superior can come to help to deal with the problem. However, instead of leaders, security personnel come only to persuade the family to leave. These midwives know that this matter cannot be handled without the appearance of leaders.*

#### 3.4.5. Theme 5: Large Physical Workload

*Unwell Symptom*: “We should be always ready for working at lunchtime of day shifts. We worry about the situation of puerperae, so we are too nervous to have lunch, which can cause dyspepsia. In addition, I have severe scapulohumeral periarthritis so that I cannot feel the breeze and be too tired.” (ID 1).

*Harmful Stimulation*: “When there is no pain-free delivery, sometimes puerperae shout loudly, which is a kind of harmful stimulation. In the meantime, we will doubt that whether contractions or any other unwell symptoms occur, which makes us worried and depressed.” (ID 9).

*Overdo the Sympathy*: “Once we induced a puerpera because the 8-month baby had hydrothorax and hydro-abdomen. Due to sympathy, we did the natural labour. Unfortunately, the puerpera died because of amniotic fluid embolism. Actually, as a midwife, overdoing the sympathy may hurt puerperae even more. Investing too much emotion may impede making a right decision.” (ID 33).

#### 3.4.6. Theme 6: Poor Working Environment

*Disharmony Relationships with Colleagues: “Instead of workloads, disharmony relationships with colleagues and leaders can drive people crazy. If you cannot get along well with your colleagues and leaders, you will suffer from work and feel frustrated.” (ID 14).*

*Unreasonable management system: ID 4 said that in their department, they have no say in many matters and anything will be decided by our leaders. She thinks this research is valuable, and they can express their hearts.*

*Leader Lack Responsibilities*: “Our leader does not have a strong sense of responsibility. When medical disputes occur, the leader will pass the buck on us. I feel frustrated and lack enthusiasm for working.” (ID 22).

*Lack the Cooperation between Doctors and Midwives*: “We do not have enough communications with doctors. If there are differences between their knowledge and our guidelines, we cannot work well with each other and may have disagreements.” (ID 28).

#### 3.4.7. Theme 7: Unbalance Between Work and Family

*Owe to Families*: “We are much busier than usual during festivals and I have already been on duty on New Year's Eve for 10 years. My dad always complains that I have not enough time to spend with them. I feel guilty and owe them so much.” (ID 31).

*Self-sacrifice: “I desire to have a second child because of the two-child policy. However, I chose to miscarry due to large pressure and workloads. I was suffering from making this choice for a long time. I would say I give up many things for my work and feel helpless (silent tears).” (ID 34).*

*Helpless: “My family does not understand me and think it is unfair for me to do such a busy work but earn the less money. When I go to work after maternity leave, they go to the hospital to defend against my situation, which has become a joke in the eyes of my colleagues. I scold myself for my powerless and feel overwhelmed.” (ID 22).*

## 4. Discussion

This research demonstrated that compassion satisfaction scored (32.64 ± 6.47), job burnout scored (27.89 ± 5.01), and secondary traumatic stress scored (26.31 ± 5.70). The scores all exceeded their critical values. The scores of all dimensions of compassion fatigue were higher than those of the mental health nurses and the oncology nurses. The compassion fatigue scores of midwives were moderate or above. The incidence is higher than that of nurses in general clinical departments studied [15–17]. The incidence of mild or above compassion fatigue among midwives was higher than nurses from common departments [17]. Most puerperae and their families lack the psychological adaptation stage for some emergencies in delivery rooms. Thus, when emergencies occur, it will be difficult for puerperae and their families to accept, and they will have extreme emotions or behaviors. These emotions, behaviors, or the matter itself will leave scares on midwives and impact their careers [18]. At the same time, when observing labor, the midwife not only bears the demands and groans caused by the mother's pain, but this kind of bad sound stimulation makes the midwife bear the greater mental and psychological pressure in addition to the safety of pregnancy and fetal life. In Rice's study [19], 35% of midwives had moderate or above compassion fatigue, which is different from the 82.13% of moderate or above compassion fatigue in this study, which may be compared with the number of births after the opening of the second child policy in China. As high-risk and elderly mothers increase, midwives need to undertake high-level and continuous maternal and child health prenatal, mid- and postnatal care services, which put midwives in stress and high-load, high-risk work conditions, also probably, the number of midwives per 1,000 population in our country is 0.05, which is much lower than that of developed countries and some developing countries. The shortage of human resources allocation on the one hand, must meet the needs of new midwifery training and learning needs for new midwifery technology and Doula services, and on the other hand, it must meet the human resource needs of the development of Doula midwifery services, which is related to the heavy workload [20].

Muliira [21] indicates in his study that midwives in the deprived areas or basic hospitals are more prone to have compassion fatigue because of poor medical environment, low wages, and the lack of social support. This research arrived at the same conclusion. Secondary and western hospitals have lower resource support, poorer medical conditions, and lower wages than other hospitals in China. Especially in western areas, the requirement of quantity of midwives is higher and the level of care for serious diseases is lower. With the demanding requirements of specialized abilities for midwives, they still cannot have sufficient chances to participate in training outside [22]. In China, obstetrics resources mainly focus on areas with a large population, leading to the unbalanced distribution of health resources [23]. This study also demonstrated that the level of midwives' compassion fatigue in tertiary hospitals was higher than specialized hospitals. The possible reasons could be that the numbers of older puerperae increases because of the childbearing policy and tertiary hospitals conduct more rescue work of serious diseases with taking more risks. Combined with the policy, it is crucial to build the talent group for grassroots health care and establish the mechanism of division and cooperation of medical institutions in integrated health care system [24]. Meanwhile, to advance the balanced development of different classes of hospitals in different areas, tertiary hospitals are encouraged to develop close relationship with secondary and basic hospitals and assist to optimize medical resources. In addition, in this study, there was a negative correlation between social support level and compassion fatigue level. Sadie [25] has examined that supports from family, friends, and organization is crucial for midwives. Lacking supports from colleagues and leaders can make midwives lack the sense of belonging [26], thus increasing repressed emotions of midwives. Some research state that insufficient social support can increase the incidence of compassion fatigue of midwives [27]. The low objective support in this study indicates that the support from social groups, organizations, family, and friends to midwives is low. The lack of support from colleagues, leaders, and teams at work, or lack of recognition and attention will make midwives feel that the working atmosphere is not harmonious, will make midwives feel double pressure from work and life, and easily cause midwives to empathize and fatigue. The low use of support means that the individual cannot perceive all aspects of support. On the one hand, it is due to the low objective support. On the other hand, it shows that the individual cannot make good use of the objective conditions brought about by objective support and cannot recognize objective support. The material and spiritual needs brought about, and the use of support is closely related to the job burnout of midwives, which also shows that individuals cannot perceive and use the support from external organizations and society and there will be numbness and burnout at work more serious.

In this research, 66.41% of midwives experienced at least three traumatic deliveries. The more traumatic deliveries they experienced, the more serious their compassion fatigue level would be. In other ways, more traumatic deliveries can make midwives lack confidence of their skills and abilities, thus producing negative emotions and inducing compassion fatigue [2]. Organizing and rationally handling childbirth traumatic events is the greatest traumatic psychological support for midwives. According to Julia's systematic reviews [25], experiencing traumatic deliveries will increase the risk of traumatic stress reactions, further forming a series of compassion fatigue symptoms such as “Sympathy price”, .that reaches a consensus with this study. Traumatic delivery can not only bring pains and trauma to midwives but also make them feel the lack of capacity for compassion increasingly, which is the primary reason of compassion fatigue [28]. When adverse childbirth events occur, puerperae and families are formidable to accept, and conflicts, or even violence, will happen. Therefore, what leaders will do to cope with this situation will impact midwives. In this research, some leaders only focus on comforting puerperae and their families and hold the midwives accountable. Whereas, some midwives who are mentally weak will get into extreme panic and anxiety if the hospital cannot handle this problem positively. Instead, there are some organizations abroad providing psychological supports and helps to those who experience traumatic deliveries, so as to ensure that they can better devote into work [29].

Pierce [30] argues that due to passive work postures and large workloads, 40% of midwives have some predictable diseases, such as lumbago caused by lumbar muscle strain and lower urinary tract symptoms (LUTS) caused by delayed micturition and stressed obesity. This contributes a lot to the increasing rate of job changes of midwives. In this study, poor sleep quality is the impact factor of compassion fatigue, and sleep disorder is one of the physical symptoms of compassion fatigue. On the one hand, some predictable diseases from working can lead to insomnia; on the other hand, puerperae always release the highest levels of oxytocin and melatonin in the night so that the most of deliveries happen in the night. This make midwives work overtime in night shifts and thus influences their physiological sleep cycle [31]. Meanwhile, because of the particularity of working environment and large workloads, midwives may have a series of unwell symptoms, such as dyspepsia, shoulder pains, palpitation, and nervousness. Such a situation can reduce the motivation of midwives and increase their physical and mental loads. Consequently, it is crucial to pour attention to both mental and physical health of midwives, so as to conduct the human-based management.

## 5. Conclusion

This research covers 3 economic areas, 12 provinces, and 57 different levels of public hospitals, thus the results are representative. This study only concentrates on midwives who are still occupied in midwifery, however, the staff turnover of midwifery keeps a high level in China. Future study can focus on resigned personnel or transferees to other departments to optimize the construction of midwife team. Meanwhile, workloads, wages, and working environment are all analyzed from the subjective point of view of midwives. It is worthwhile, make them more quantifiable in future research to make data more objective.

## Figures and Tables

**Table 1:** Numbers of investigated hospitals.

Area/Province	Hospital(numbers, *n* = 57)			Midwives [Number (percentage %)]
	Secondary	Tertiary	Specialized	
Eastern area				170 (33.01)
Hebei	2	2	1	40 (7.77)
Jiangsu	1	2	1	45 (8.74)
Guangdong	2	2	2	43 (8.35)
Shandong	1	2	1	42 (8.15)
Central area				170 (33.01)
Hubei	2	2	1	47 (9.13)
Henan	2	2	1	46 (8.93)
Jiangxi	1	2	1	40 (7.77)
Anhui	2	2	1	37 (7.18)
Western area				175 (33.98)
Gansu	2	2	1	49 (9.51)
Qinghai	2	1	1	41 (7.96)
Chongqing	2	2	1	45(8.74)
Guizhou	2	2	1	40 (7.77)

**Table 2:** Single factor analysis of compassion fatigue among midwives.

Project	Degree of compassion fatigue		Statistics	*P* value
	None and mild	Moderate and above		
Level of hospital			12.040^1)^	0.002
Secondary	15 (8.98)	152 (91.02)		
Tertiary	29 (16.86)	143 (83.14)		
Specialized	48 (27.27)	128 (72.73)		
Area			18.860^1)^	< 0.001
Eastern	61 (23.78)	129 (76.22)		
Central	38 (21.25)	132 (78.75)		
Western	15 (8.58)	160 (91.42)		
Age			32.601^2)^	< 0.001
20~	35 (38.89)	55 (61.11)		
2 6~	26 (13.54)	166 (86.46)		
3 1 ~	15 (10.71)	125 (89.28)		
> 3 5	15 (16.13)	78 (83.87)		
Marriage situation				
Unmarried	47 (34.06)	91 (65.94)	45.560^1)^	< 0.001
Married	44 (12.72)	302 (87.28)		
Divorced	2 (6.45)	29 (93.55)		
Sleep quality			24.760^2)^	< 0.001
Normal	34 (31.78)	73 (68.22)		
Occasional insomnia	37 (16.89)	182 (83.11)		
Frequent insomnia	12 (7.95)	139 (92.05)		
Children situation			59.646^2)^	< 0.001
None	53 (35.57)	96 (66.43)		
Infant	18 (11.18)	143 (88.81)		
School-age	6 (5.04)	113 (94.96)		
Junior school and above	17 (19.77)	69 (80.23)		
Experiences of traumatic delivery			76.138^2)^	< 0.001
0	29 (60.42)	19 (39.58)		
1~	14 (11.20)	111 (88.80)		
3~	17 (11.41)	132 (88.59)		
> 5	13 (6.74)	180 (93.26)		
Job satisfaction			44.039^2)^	< 0.001
Very satisfied	4 (40.00)	6 (60.00)		
Satisfied	47 (37.90)	77 (62.10)		
Ordinary	29 (10.43)	249 (89.57)		
Very unsatisfied	6 (5.83)	97 (94.17)		
Whether workload is too large			13.656^2)^	0.004
Yes	36 (14.46)	213 (88.54)		
Ordinary	49 (20.08)	195 (79.92)		
No	3 (13.64)	19 (86.36)		
Whether to like work environment			20.753^2)^	< 0.001
Yes	47 (27.81)	122 (72.19)		
Ordinary	32 (12.17)	231 (87.83)		
No	4 (4.82)	79 (95.18)		
Social support level			113.154^2)^	< 0.001
Low	12 (7.36)	151 (92.64)		
Medium	28 (9.89)	255 (90.11)		
High	43 (62.31)	26 (37.69)		

Note. 1: *χ*2 value; 2: *χ*2 value (Kruskal–Wallis).

**Table 3:** Zero-level analysis of two-level variance components.

Parameter	Estimate	Standard error	*P* value
Fixed effect			
Intercept	1.7768	0.1722	< 0.0001
Random effect			
Level 2 variance	0.6895	0.2931	0.0093
Level 1	1		

**Table 4:** Independent variables assignment table.

Variables	Value
Compassion fatigue	None and mild = 0, Moderate and above = 1
Hospital Level	Specialized hospital (*Z*1 = 0, *Z*2 = 0), Secondary (*Z*1 = 1, *Z*2 = 0), Tertiary (*Z*1 = 0, *Z*2 = 1)
Area	Eastern area (*Z*1 = 0, *Z*2 = 0), Central area (*Z*1 = 1, *Z*2 = 0), Western area (*Z*1 = 0, *Z*2 = 1)
Age	20~ (*Z*1 = 0 , *Z*2 = 0, *Z*3 = 0), 26~ (*Z*1 = 1, *Z*2 = 0, *Z*3 = 0), 31~ (Z_1_ = 0, *Z*2 = 1, *Z*3 = 0), >35 (*Z*1 = 0, *Z*2 = 0, *Z*3 = 1)
Marriage situation	Unmarried (*Z*1 = 0, *Z*2 = 0), Married (*Z*1 = 1, *Z*2 = 0), Divorced (*Z*1 = 0, *Z*2 = 1)
Sleep quality	Normal (*Z*1 = 0, *Z*2 = 0), Occasional insomnia (*Z*1 = 1, *Z*2 = 0), Frequent insomnia (*Z*1 = 0, *Z*2 = 1)
Children situation	None (*Z*1 = 0, *Z*2 = 0, *Z*3 = 0), Infant (*Z*1 = 1, *Z*2 = 0, *Z*3 = 0), School-age (*Z*1 = 0, *Z*2 = 1, *Z*3 = 0), Junior school and above (*Z*1 = 0, *Z*2 = 0, *Z*3 = 1)
Experiences of traumatic delivery	0 (*Z*1 = 0, *Z*2 = 0, *Z*3 = 0), 1~2 (*Z*1 = 1, *Z*2 = 0, *Z*3 = 0), 3~5 (*Z*1 = 0, *Z*2 = 1, *Z*3 = 0), >5 (*Z*1 = 0, *Z*2 = 0, *Z*3 = 1)
Job satisfaction	Very satisfied (*Z*1 = 0, *Z*2 = 0, *Z*3 = 0), Satisfied (*Z*1 = 1, *Z*2 = 0, *Z*3 = 0), Ordinary (*Z*1 = 0, *Z*2 = 1, *Z*3 = 0), Very unsatisfied (*Z*1 = 0, *Z*2 = 0, *Z*3 = 1)
Whether workload is too large	Yes (*Z*1 = 0, *Z*2 = 0), Medium (*Z*1 = 1, *Z*2 = 0), No (*Z*1 = 0, *Z*2 = 1)
Whether to like the working environment	Yes (*Z*1 = 0, *Z*2 = 0), Medium (*Z*1 = 1, *Z*2 = 0), No (*Z*1 = 0, *Z*2 = 1)
Social support level	Low (*Z*1 = 0, *Z*2 = 0), Medium (*Z*1 = 1, *Z*2 = 0), High (*Z*1 = 0, *Z*2 = 1)

**Table 5:** Multilevel statistical models analysis results of impact factors of midwives' compassion fatigue.

Independent variables	Estimated value	Standard error	*P* value	OR Value (95% CI)
Intercept	3.2069	1.3623	0.009	—
Level 2 (Hospital)				
Hospital level (Specialized)				1
Secondary	-0.2361	1.2622	0.8517	0.790
Tertiary	-4.4947	1.1901	0.0002	0.011
Area (East)				1
Central	-1.4854	1.0147	0.1440	0.226
Western	-3.3545	0.8654	0.0001	0.035
Level 1 (Individual)				
Sleep quality (normal)				1
Occasional insomnia	-0.01376	0.9014	0.9878	0.986
Frequent insomnia	0.3906	1.4038	0.7809	1.478
Children situation (None)	0.1325	1.4651	0.9280	1.142
Infant				1
School-age	1.1807	1.1457	0.3033	3.257
Junior school and above	2.5925	2.2225	0.2441	13.363
Experiences of traumatic delivery (0)	0	.	.	1
1~2	1.4194	1.0684	0.1847	1.805
3~5	1.2981	1.5081	0.3899	2.708
>5	-0.576	1.2398	0.6425	1
Whether to like working environment (Yes)	0	.	.	4.134
Medium	0.5903	0.6793	0.3853	3.662
No	0.9961	0.8083	0.2185	0.562
Social support level (Low)	0	.	.	1
Medium	1.7773	0.9261	0.0556	5.914
High	1.4653	0.9415	0.1203	4.329

**Table 6:** Basic information of 34 midwives.

Coding	Interview method	Age	Title grade	Marriage situation	Children situation	years	Hospital level	Province	ETD	CF degree
M1	Video	29	Junior	Married	School-age	3	Secondary	Shandong	3	Moderate
M2	Video	34	Junior	Married	Primary school	7	Tertiary	Shandong	> 5	Moderate
M3	Face-to-face	29	Junior	Married	School-age	6	Tertiary	Shandong	3	Moderate
M4	Video	27	Junior	unmarried	None	4	Specialized	Shandong	4	Moderate
M5	Video	29	Junior	Married	None	6	Secondary	Shandong	3	Severe
M6	Face-to-face	39	Middle	Married	Junior school	17	Tertiary	Hebei	> 5	Moderate
M7	Video	26	Junior	unmarried	None	2	Tertiary	Hebei	2	Moderate
M8	Video	35	Junior	Married	Junior school	15	Secondary	Hebei	> 5	Moderate
M9	Face-to-face	34	Junior	Married	Primary school	12	Specialized	Hebei	> 5	Moderate
M10	Video	28	Junior	Married	School-age	5	Secondary	Hebei	3	Severe
M11	Face-to-face	37	Junior	Divorced	Primary school	27	Secondary	Henan	> 5	Mild
M12	Face-to-face	38	Middle	Married	University	28	Secondary	Henan	> 5	Moderate
M13	Face-to-face	32	Middle	Married	School-age	10	Specialized	Henan	> 5	Moderate
M14	Face-to-face	34	Junior	Married	School-age	12	Secondary	Henan	4	Moderate
M15	Face-to-face	30	Junior	Married	School-age	6	Tertiary	Henan	3	Moderate
M16	Face-to-face	30	Junior	Married	School-age	8	Tertiary	Henan	4	Moderate
M17	Face-to-face	32	Junior	Married	Primary school	4	Tertiary	Hubei	> 5	Moderate
M18	Face-to-face	45	Middle	Married	University	27	Specialized	Hubei	> 5	Moderate
M19	Face-to-face	28	Junior	unmarried	None	4	Secondary	Hubei	4	Severe
M20	Video	39	Middle	Married	University	19	Tertiary	Hubei	> 5	Severe
M21	Video	34	Junior	Married	Primary school	12	Tertiary	Hubei	> 5	Moderate
M22	Face-to-face	33	Junior	Married	School-age	9	Secondary	Hubei	4	Moderate
M23	Face-to-face	34	Middle	Married	Primary school	5	Tertiary	Chongqing	4	Severe
M24	Face-to-face	31	Middle	Married	Primary school	10	Secondary	Chongqing	3	Moderate
M25	Face-to-face	31	Junior	Married	School-age	9	Tertiary	Chongqing	3	Moderate
M26	Face-to-face	26	Junior	unmarried	None	5	Specialized	Chongqing	4	Moderate
M27	Face-to-face	29	Junior	Married	School-age	5	Secondary	Chongqing	3	Moderate
M28	Face-to-face	28	Junior	Married	School-age	5	Secondary	Chongqing	4	Moderate
M29	Video	29	Junior	Married	Primary school	7	Tertiary	Gansu	> 5	Moderate
M30	Video	33	Middle	Married	Junior school	12	Tertiary	Gansu	> 5	Moderate
M31	Video	37	Junior	Married	Junior High school	27	Secondary	Gansu	> 5	Moderate
M32	Face-to-face	24	Junior	unmarried	None	2	Tertiary	Gansu	2	Moderate
M33	Video	34	Junior	Married	Primary school	10	Secondary	Gansu	3	Moderate
M34	Video	29	Junior	Married	School-age	5	Specialized	Gansu	2	Severe

Note: EBT(Experienced birth trauma).

## Data Availability

The data used to support the findings of this study are available from the corresponding author upon request.
